# Effect of Atropine Eye Drops Combined with VR-Based Binocular Visual Function Balance Training for Prevention and Control of Juvenile Myopia

This article has been retracted.

**DOI:** 10.1155/2022/4159996

**Published:** 2022-09-13

**Authors:** Yuping Shi

**Affiliations:** Chengdu Aier Eye Hospital, Chengdu 610041, Sichuan, China

## Abstract

**Purpose:**

This study mainly analyzes the efficacy of 0.01% atropine eye drops (low-dose atropine (LDA)) combined with virtual reality (VR)-based binocular visual function (BVF) balance training in the prevention and control of juvenile myopia.

**Methods:**

One hundred and thirty-six juvenile myopia patients admitted between November 2018 to November 2021 were selected, including 76 cases (research group) receiving LDA + VR-based BVF balance training and 60 cases (control group) treated by LDA intervention alone. Visual acuity (VA; naked vision), ocular parameters (pupil diameter (PD), axial length (AXL), and diopter), intraocular pressure (IOP), accommodation facility, clinical efficacy, and incidence of adverse reactions were observed, compared, and analyzed in both groups.

**Results:**

After analysis, it was found that the research group showed significantly higher naked vision and PD while statistically lower *D* after intervention than the corresponding preinterventional parameters than the control group. While AXL showed no statistical difference between the groups and within groups. The IOP also differed insignificantly between groups, but the post-treatment accommodation facility was better in the research group compared with the baseline (before treatment) and control group. In terms of curative effects, an obviously higher total effective rate was determined in the research group. In addition, the two groups showed no significant difference in the incidence of adverse reactions.

**Conclusions:**

LDA + VR-based BVF balance training deserves clinical popularization, as it can prevent and control myopia among teenagers, with better adjusting effects on eye function and certain safety.

## 1. Introduction

Myopia, the main inducement of visual impairment and blindness, shows a growing incidence [1]. A higher risk of myopia is associated with factors such as women, teenagers, impaired eyesight of parents, less outdoor activities, and more time spent watching videos [2, 3]. Statistics show that myopia, as a major public health issue of modernization, is expected to affect 49.8% of the global population in 2050, with a possible prevalence of up to 90% in East Asia and 20% of the cases evolving into high myopia [4]. Myopia-induced visual impairment may lead to high myopia-associated complications, including cataract, glaucoma, retinal detachment, myopic macular degeneration, and choroidal neovascularization [5, 6], which may bring inconvenience to the study and life for adolescent students and cause a great socio-economic burden [7]. Therefore, it is of great implications to explore intervention measures for the prevention and control of myopia among teenagers to alleviate juvenile myopia and avoid high myopia.

At present, the major goal of myopia treatment is to slow down the progression of high myopia, with the primary treatment strategies covering medication, vision training, glasses, orthokeratology, and laser surgery [8, 9]. The focus of this study is to explore effective prevention and control measures for myopia from the perspectives of drugs and visual training. Tropine, in essence, is a nonselective muscarinic receptor antagonist. Eye drops made from it are often used not only as an intervention for children's progressive myopia, but also for the treatment of pediatric eye diseases such as cycloplegia, amblyopia, and strabismus [10]. And, given the allergic reactions to the eyes, atropine eye drops is often given at a low dose to myopic children [11]. Studies have shown that 0.01% atropine eye drops (low-dose atropine (LDA)) has no significant adverse effects on children's optical quality, with better therapeutic safety than 0.05% atropine eye drops [12]. In terms of visual training, virtual reality (VR)-based binocular visual function (BVF) balance training is a kind of stereoscopic perception training for patients by wearing VR visual training glasses. It helps patients fully exercise their ciliary muscles from visual training, scenery, movies, games, experience halls and other sectors, thus achieving the effect of preventing myopia and relieving visual fatigue [13].

There are currently few related studies investigating the clinical effect of LDA combined with VR-based BVF balance training on the prevention and control of juvenile myopia. Accordingly, this study conducted relevant clinical analysis, aiming at providing a new reliable basis for the prevention and control of juvenile myopia.

## 2. Data and Methods

### 2.1. Baseline Information

This research selected 136 cases of juvenile myopia treated between November 2018 and November 2021 and grouped them as follows according to different treatment modalities: a research group (*n* = 76) treated by LDA + VR-based BVF balance training, and a control group (*n* = 60) given only LDA. This research has obtained approval from the Chengdu Aier Eye Hospital's Ethics Committee and informed consent from all subjects.

### 2.2. Inclusion and Exclusion Criteria

Adolescents who met the diagnostic criteria for myopia [9], with no other eye diseases as indicated by ophthalmic examinations, no parental history of high myopia, good compliance, and regular reviews as required were enrolled.

Teenagers who had precious eye surgery or eye trauma, atropine allergies or medication contraindications, use of atropine eye drops, and orthokeratology to control myopia, or ocular organic diseases like strabismus, amblyopia, and glaucoma were excluded.

### 2.3. Treatment Methods

Before treatment, all patients underwent ocular examinations to examine their naked vision, ocular parameters (pupil diameter (PD), axial length (AXL), and diopter (D)), intraocular pressure (IOP), and accommodation facility to check for diseases of both the anterior segment and fundus.

The control group was given LDA (Topfond Pharmaceutical, H41020291) once a day, one drop at a time. The hands should be cleared before applying the medicine, and it is advisable to administer the medicine at 9–10 pm and press the lacrimal sac for about 3 minutes after drug use. After that, patients can do homework and read books for a short period of time but cannot use electronic products.

The research group was given LDA + VR-based BVF balance training. VR balance training is divided into visual training, scenery, movies, games, experience, etc. When the patient wears VR glasses (More Light Technology, Co., Ltd.), the eyes can alternate far and near, left and right, up and down, and rotate 360°. In this way, the eyes can change the angle, direction, and sight distance in the virtual world, and exercise the ciliary muscles in an all-round way, so as to gradually restore the mutated organs to normal, thus preventing myopia and relieving eye fatigue. The training methods are as follows: 4 training items were carried out every day, with the first two in the morning and the last two in the afternoon. The interval between morning and afternoon training was at least 2 hours, and each training item was performed for 10 minutes (5 minutes for left and right eyes, respectively) with a 10-minute break between items. Fatigue-prone patients with astigmatism exceeding 200° could adopt the method of low intensity and high frequency, with each training items lasting for 5 minutes and 4–6 items every day. During the holidays, the number of training sessions could be increased to three times a day, which were conducted in the morning, middle, and evening, respectively, with a total of 6 items. The following points should be noted during treatment: (1) keep training every day; (2) avoid training in a state of fatigue. Patients were reviewed monthly for visual acuity (VA) and eye position so that training regimens could be adjusted accordingly based on recovery. In addition, patients used LDA, one drop, each time before going to bed and pressed on the lacrimal sac for about 3 minutes. The treatment period of both the groups was 6 months.

### 2.4. Detection Methods

1. VA: patients' naked vision, when the ciliary muscle was fully paralyzed after correcting VA by insertion and computer optometry, was recorded before and 6 months after intervention
2. Ocular parameters: after measurement of pupil diameter by using a Pentacam anterior segment analyzer (Shanghai Hanfei Medical Equipment Co., Ltd.), corneal topography was used for remeasurement in the same dark room. The average value was obtained after three measurements. AXL was determined by an IOL Master, and *D* was measured using 1% compound Tropicamide eye drops (Beijing Shuanghe Modern Medical Technology Co., Ltd., H11021793) for cycloplegia. The abovementioned eye parameters were measured before and 6 months after the intervention.
3. IOP and accommodation facility: the IOP was measured using a noncontact tonometer (Shanghai Jumu Medical Equipment Co., Ltd., c0081), and the accommodation facility was measured within 1 min by using corrective eyeglasses and lens Dflipper and flipper for hyperopia. The IOP and accommodation facility of the two groups were measured and compared before and after 6 months of treatment.
4. Therapeutic effect: patients were considered to be markedly effective if the *D* remained stable, effective if the *D* increased within 0.75D, and ineffective if the *D* increased more than 0.75D after 6 months of treatment. The markedly effective, effective, and ineffective cases of the two groups were recorded, and the total effective rate was calculated. The total effective rate was the percentage of the sum of the effective and effective cases in the total cases.
5. Safety: adverse events (AEs) such as photophobia, near-vision difficulties, and glare were recorded and analyzed, and the total incidence of AEs was calculated

### 2.5. Statistical Processing

SPSS19.0 and Graphpad Prism 7 were utilized for data processing and visualization, respectively. ($\bar{x}\pm s$) and (n/%) were used to represent measurement data and count data, respectively. The independent sample *t*-test was used to analyze the measurement data between groups, the *χ*^2^-test to analyze the count data between groups, and the paired *t*-test to analyze the measurement data between two time points. Analysis results with *P* < 0.05 were statistically significant.

## 3. Results

### 3.1. Baseline Information

As shown in Table 1, the two groups showed nonsignificant differences in baseline data in terms of age, sex, only child, time spent outdoors, sleeping time, family history of myopia, education level of primary caregivers, and residence (*P* > 0.05).

### 3.2. VA in Both Groups

We tested naked vision in both cohorts to evaluate the influences of the two interventions on patients' VA (Figure 1). We found no statistical difference between groups in the naked vision before treatment (*P* > 0.05); a marked improvement was observed in naked vision in both cohorts after treatment, with a more significant improvement in the research group (*P* < 0.05).

### 3.3. Ocular Parameters in Both Groups

The PD, AXL, and *D* of the two cohorts were measured (Figure 2). The abovementioned three ocular parameters of the two groups showed no significant difference prior to treatment (*P* > 0.05). The PD of both cohorts increased statistically after intervention (*P* < 0.05), and the *D* decreased markedly (*P* < 0.05), while the AXL showed no significant difference before and after intervention (*P* > 0.05). The research group had a higher PD and a lower *D* than the control group (*P* < 0.05), while the AXL was similar in the two groups (*P* > 0.05).

### 3.4. IOP and Accommodation Facility in Both Groups

No statistical difference was observed between the two groups in pretreatment IOP and accommodation facility (*P* > 0.05), nor was there any difference in pretreatment and post-treatment IOP (*P* > 0.05). While the accommodation facility of both cohorts increased markedly after intervention (*P* < 0.05), with higher accommodation facility in the research group compared with the control group (*P* < 0.05) as shown in Figure 3.

### 3.5. Clinical Efficacy of the Two Groups

We evaluated patients' clinical outcomes to validate the effectiveness of both interventions (Table 2). The results revealed a higher total effective rate in the research group (92.10%) compared with the control group (80.00%), with a statistical significance (*P* < 0.05).

### 3.6. Incidence of AEs in Both Groups

We analyzed the incidence of AEs in both groups to assess the safety of both interventions (Table 3). The results showed a nonsignificant difference between the research group and control group in AEs (3.95% VS 8.33%, *P* > 0.05).

## 4. Discussion

Myopia is a global epidemic of ocular vision disorders caused by the interaction of multiple factors, which is common in teenagers [14]. Finding an effective, safe, and reliable therapy to alleviate myopia progression is critical to improving VA in adolescents.

Current interventions for the prevention and control of myopia include orthokeratology, dietary supplementation of omega-3 polyunsaturated fatty acids (*ω*-3 PUFA), and increasing outdoor time. Orthokeratology has been shown to improve eye regulation in children to prevent and control myopia; *ω*-3 PUFA protects VA in adult workers by reducing job-related choroidal blood perfusion, while increasing outdoor time prevents myopia primarily by reducing axial length changes [15–17]. The report of myopia prevention and control in this study mainly focuses on atropine eye drops and VR-based BVF balance training. The use of atropine eye drops has been proven effective in improving myopia in a series of studies, but there is a certain risk of complications [17–19]. LDA has been recommended by the American Academy of Ophthalmology to prevent and control myopia [20]. The VR-based balance training of BVF is realized with the use of head-mounted displays, allowing teenagers to change the angle, direction, and visual distance of their eyes in the virtual world, and exercising their ciliary muscles in an all-round way, so as to gradually restore their vision with the recovery of the visual organ function [21]. In our study, 136 adolescent myopia patients were included, of which 76 cases in the research group received LDA + VR-based BVF balance training, and 60 cases in the control group only received LDA. Our research data showed that both vision repair interventions had significant effects on the naked vision improvement of juvenile myopia patients, but LDA + VR-based BVF balance training contributed to a better improved naked VA level in the research group, indicating that the combined intervention was superior to LDA alone in improving VA. Žiak et al. [21] pointed out that amblyopia patients had significantly improved best corrected VA and stereoscopic vision after receiving VR-based BVF balance training, suggesting the effectiveness of this treatment in improving patients' VA level, similar to our research results.

The ocular parameters of all participants were also analyzed. The results showed that research group had significantly better PD and *D* under the joint intervention, but the AXL had no significant difference with the control group, which is consistent with the findings of Jethani et al. [22]. In addition, IOP showed no significant difference between groups and within the groups before and after treatment, indicating that neither of the two treatment methods would increase the IOP of patients. Yu et al. [23] reported that atropine eye drop intervention did not cause high IOP in myopic children, nor atropine eye drop intervention under different cumulative did, which was consistent with our research results. And, although some studies have shown that increased IOP is a short-term side effect of atropine, another prospective study also confirmed that atropine eye drops did not cause increased IOP within one year in myopic patients [24]. However, we found more prominent effects of the combined therapy on improving the eye accommodation facility of juvenile myopia patients. The reason may be related to the synergistic effect of LDA + VR-based BVF balance training intervention on the alleviation of myopia in adolescents. The combination of the two can effectively inhibit the further progression of myopia, improve the VA level of patients, and delay the increase of AXL and *D*, thus increasing the PD of subjects. Moreover, the patient's ciliary muscles were fully trained under the VR-based BVF balance training, which further improved the ciliary muscle movement rate, amplitude and muscle strength, enhanced blood supply, and significantly improved the eye focus, contributing to an effectively enhanced accommodation facility of the subject's eyes without increasing IOP. Similarly, Huang et al. [25] confirmed that VR-based BVF balance training can effectively repair the eye accommodation lag of myopia patients and improve their ocular accommodation function. Furthermore, we evaluated the clinical efficacy and safety of the two treatment strategies. The data showed a significant difference in the total effective rate between the research group and control group (92.10% VS 80.00%), while there was no statistical significance in the incidence of AEs (3.95% VS 8.33%). This shows that the prevention and control of juvenile myopia with VR-based BVF balance training is not only effective, but also safe, which is similar to the research results of Larkin et al. [26].

The novelties of this study are as follows: (1) through the analysis of naked vision and efficacy, it is confirmed that LDA combined with VR-based BVF balance training can effectively protect young people's vision; (2) the specific effects of the joint intervention were analyzed from the perspectives of ocular parameters such as PD, AXL, and *D*, as well as IOP and accommodation facility; (3) it has been confirmed from the safety aspect that the combination therapy has certain safety and will not increase the incidence of AEs. The abovementioned multidimensional analysis provides an optimal choice for the prevention and control of myopia in adolescents. Still, there are some limitations that need further consideration. First, risk factors for high myopia in adolescents have not been analyzed, and supplementing this analysis may help improve prevention and control strategies for myopia. Second, the study time is short, and extension of the research time can further provide insight into the effectiveness of long-term interventions and the clinical effect after stopping the intervention for a period of time.

## 5. Conclusion

To sum up, LDA combined with VR-based BVF balance training has definite efficacy in the prevention and control of juvenile myopia, which can significantly improve the VA level of patients without increasing the incidence of AEs, with a certain clinical promotion value.

## Figures and Tables

**Figure 1:** Naked vision in both groups. Note: ^*∗*^ represents *P* < 0.05 compared with the level before treatment; ^#^ represents *P* < 0.05 compared with the control group.

**Figure 2:** Ocular parameters in both groups. (a) The pupil diameter of the research group after intervention was significantly higher than that before intervention than the control group. (b). There was no significant difference in the axial length between and within the two groups. (c). The diopter of the research group was significantly lower after intervention than before intervention than the control group. Note: compared with before treatment, ^*∗*^*P* < 0.05; compared with the control group, ^#^*P* < 0.05.

**Figure 3:** Intraocular pressure and accommodation facility in both groups. (a). There was no significant difference in intraocular pressure between and within the two groups. (b). The accommodation facility of the research group increased significantly after intervention and was significantly higher than that of the control group. Note: ^*∗*^ represents *P* < 0.05 compared with the level before treatment; ^#^ represents *P* < 0.05 compared with the control group.

**Table 1:** Baseline data of two groups of patients (*n* (%), mean ± SEM).

Factors	Control group (*n* = 60)	Research group (*n* = 76)	*χ* ^2^/*t*	*P*
Age (years)	16.05 ± 2.09	16.42 ± 3.05	0.802	0.424

Sex			0.055	0.815
Male	32 (53.33)	39 (51.32)		
Female	28 (46.67)	37 (48.68)		

Only child			0.936	0.333
Yes	25 (41.67)	38 (50.00)		
No	35 (58.33)	38 (50.00)		

Time spent outdoors (hours/weeks)			2.821	0.244
<7	16 (26.67)	30 (39.47)		
7–17	26 (43.33)	30 (39.47)		
≥14	18 (30.00)	16 (21.06)		

Sleep time (hours/days)			1.161	0.560
<7	6 (10.00)	12 (15.79)		
7–9	36 (60.00)	45 (59.21)		
≥9	18 (30.00)	19 (25.00)		

Family history of myopia			1.432	0.232
Yes	12 (20.00)	22 (28.95)		
No	48 (80.00)	54 (71.05)		

Education level of primary caregivers			0.590	0.442
High school and below	34 (56.67)	48 (63.16)		
High school or above	26 (43.33)	28 (36.84)		

Residence			0.183	0.669
Urban areas	27 (45.00)	37 (48.68)		
Rural areas	33 (55.00)	39 (51.32)		

**Table 2:** Clinical efficacy of the two groups of patients.

Classification	Control group (*n* = 60)	Research group (*n* = 76)	*χ* ^2^	*P*
Markedly effective	30 (50.00)	49 (64.47)	—	—
Effective	18 (30.00)	21 (27.63)	—	—
Ineffective	12 (20.00)	6 (7.90)	—	—
Total effective rate (%)	48 (80.00)	70 (92.10)	4.279	0.039

**Table 3:** Incidence of adverse events.

Classification	Control group (*n* = 60)	Research group (*n* = 76)	*χ* ^2^	*P*
Photophobia	2 (3.33)	2 (2.63)	—	—
Near-vision difficulties	2 (3.33)	1 (1.32)	—	—
Glare	1 (1.67)	0 (0.00)	—	—
Incidence of adverse events	5 (8.33)	3 (3.95)	1.165	0.280

## Data Availability

The labeled dataset used to support the findings of this study are available from the corresponding author upon request.
